The article "Functional Mitral Stenosis Resulting in Recurrent Flash Pulmonary Edema: A Case Report of an Atypical Complication of Streptococcus viridans Endocarditis" was published in 2023. Journal: Cureus.

# Functional Mitral Stenosis Resulting in Recurrent Flash Pulmonary Edema: A Case Report of an Atypical Complication of Streptococcus viridans Endocarditis

**DOI:** 10.7759/cureus.38670

**Published:** 2023-05-07

**Authors:** Akash Patel, Jaimin Patel

**Affiliations:** 1 Department of Medicine, Graduate Medical Education, Methodist Dallas Medical Center, Dallas, USA

**Keywords:** mitral valve vegetation, valvular heart failure, endocarditis, functional mitral stenosis, streptococcus viridans

## Abstract

Infective endocarditis (IE) can present with a wide variety of clinical signs and symptoms, making it difficult to diagnose. Recognizing risk factors such as congenital heart disease, intravenous drug use, and prosthetic heart valves can encourage early testing with blood cultures and echocardiography, leading to prompt diagnosis and treatment with antibiotics. Despite early detection and treatment, IE can still result in permanent damage of the affected heart valves, most commonly resulting in valvular regurgitation and signs and symptoms of heart failure. Clinicians must maintain a high index of suspicion as prompt diagnosis and treatment are essential to prevent morbidity and mortality. Valvular stenosis as a result of IE, unlike valvular regurgitation, is extremely rare and has only been described a handful of times in literature. We present a unique case of *Streptococcus viridans* IE resulting in functional mitral stenosis and recurrent flash pulmonary edema in an elderly female who had recently undergone a dental cleaning procedure.

## Introduction

Infective endocarditis is a rare but potentially lethal condition that can present with a wide variety of non-specific symptoms. Early detection is key in preventing morbidity and mortality, as delays in diagnosis and treatment can lead to irreversible damage to cardiac structures. Despite early intervention, one-year mortality rates remain near 40% [1]. Valvular regurgitation is widely recognized as a late complication of infective endocarditis and is even included in the modified Duke criteria as a major clinical criteria for diagnosis [2]. Valvular stenosis, unlike regurgitation, is not commonly associated with infective endocarditis but can result in similar symptoms when present. Here, we present a case of recurrent flash pulmonary edema from functional mitral stenosis in an elderly woman with *Streptococcus viridans* endocarditis.

## Case presentation

A 79-year-old Caucasian female with a past medical history of asthma, aortic stenosis status post transcatheter aortic valve replacement, hypertension, hyperlipidemia, and a remote history of lung adenocarcinoma status post lobectomy presented to the emergency department with shortness of breath, wheezing, productive cough with clear sputum, and lower extremity swelling. Her symptoms started one month ago and were progressively worsening. She denied fevers, chills, weight loss, hemoptysis, skin lesions, chest pain, or palpitations. She had recently been admitted to the hospital with similar symptoms and was diagnosed with an acute asthma exacerbation. After being discharged, she reported having to sleep in a recliner due to orthopnea. Her primary care physician referred her to the emergency department for further evaluation.

The article "Functional Mitral Stenosis Resulting in Recurrent Flash Pulmonary Edema: A Case Report of an Atypical Complication of Streptococcus viridans Endocarditis" was published in 2023. Journal: Cureus.

On initial evaluation, the patient’s vital signs were notable for SpO2 of 88% on room air, heart rate of 146, respiratory rate of 24, and a temperature of 97.9 ℉. Her SpO2 improved to 94% on 4L nasal cannula. Physical exam revealed an irregular heart rhythm, no heart murmurs, inspiratory and expiratory wheezing with bibasilar rales, elevated JVP to the angle of the mandible, and 1+ pitting edema in bilateral lower extremities. Labs were notable for an elevated white blood cell count with normal procalcitonin, NT-proBNP, and troponin levels, as seen in Table 1.

**Table 1:** Lab values on admission.

Lab Test	Patient Value	Normal Values
White blood cell count	12.3 x 10^3^/uL	3.8-11 x 10^3^/uL
Procalcitonin	0.25 ng/mL	≤0.25 ng/mL
NT-proBNP	170 pg/mL	≤1,800 pg/mL
Troponin	<0.012 ng/mL	<0.012 ng/mL

COVID and influenza testing were negative. Chest X-ray was notable for increasingly prominent interstitial markings and bilateral pleural fluid. CT angiogram did not show any evidence of pulmonary embolism or masses. Her EKG revealed atrial fibrillation with a rapid ventricular response.

The patient was admitted for acute hypoxic respiratory failure secondary to volume overload in the setting of atrial fibrillation with a rapid ventricular response. Cardiology and Pulmonology were consulted. She was started on empiric ceftriaxone and azithromycin for the treatment of community-acquired pneumonia as well as beta-blockers and diuretics for atrial fibrillation and pulmonary edema, respectively. A transthoracic echocardiogram was ordered and was notable for a left ventricular ejection fraction of 60%-65%, Grade I diastolic dysfunction, a severely dilated left atrium, and moderate mitral stenosis. There was no evidence of pericardial effusion. Over the next few days, two sets of blood cultures showed no growth, her white blood cell count normalized, and she converted to normal sinus rhythm; however, her oxygen requirements continued to escalate despite aggressive treatment with diuretics. On day six of her admission, she was requiring 24 liters of supplemental oxygen at 80% FiO2 to maintain adequate oxygen saturation. 

The article "Functional Mitral Stenosis Resulting in Recurrent Flash Pulmonary Edema: A Case Report of an Atypical Complication of Streptococcus viridans Endocarditis" was published in 2023. Journal: Cureus.

On day seven of her hospitalization, she became febrile with a temperature of 101.5 ℉. Repeat blood cultures were ordered, and grew *Streptococcus viridans*. Infectious Diseases was consulted, and after further investigation, it was revealed that the patient had undergone a dental cleaning procedure several weeks before this admission. She was empirically started on vancomycin and later transitioned to ceftriaxone once antibiotic sensitivities had resulted. Due to concerns about infective endocarditis, the decision was made to pursue transesophageal echocardiography. This revealed a large irregular, cystic gelatinous mass measuring 3 cm x 3 cm attached to the posterior leaflet of the mitral valve, as exhibited in Figure 1.

**Figure 1:** Image from transesophageal echocardiogram showing a large vegetation (yellow asterisk) attached to the posterior leaflet of the mitral valve.

The mass was noted to move in and out of the mitral valve orifice and, at times, completely block it causing functional mitral stenosis and subsequent flash pulmonary edema, as exhibited in Figure 2.

**Figure 2:** Image from transesophageal echocardiogram showing blockage of the mitral valve orifice (green lines) by a large vegetation (yellow asterisk) during atrial contraction.

Cardiothoracic Surgery was consulted, and on day 14 of her admission, the patient underwent surgical mitral valve replacement. Pathology from the mitral valve vegetation showed scant necrotic fibrous tissue and multiple calcifications in a background of abundant fibrin with acute inflammation consistent with infective endocarditis. Of note, pathology also showed benign mitral valve tissue with acute inflammation as well as invasive, moderately differentiated adenocarcinoma consistent with lung primary in the pericardium and pericardial fat. 

The patient remained intubated post-operatively and was transferred to the ICU for higher level of care. She had a prolonged ICU course complicated by pneumonia and multiple re-intubations. After several unsuccessful extubation attempts, the patient and her family decided to withdraw care, and the patient passed away on day 23 of her admission.

## Discussion

Infective endocarditis (IE) is a rare condition resulting in inflammation and colonization of the endocardium and/or heart valves by microorganisms. It is estimated to have a yearly incidence of 3 to 10 cases per 100,000 people, with a male to female ratio of approximately two to one [1]. The in-hospital mortality rate is estimated to be 18%, with a one-year mortality rate of 40% [1]. Elderly patients ages 65 and older are more likely to develop IE. Risk factors include a history of congenital heart disease, intravenous drug use, and prosthetic heart valves. Rheumatic heart disease was once a major risk factor for IE, but it now contributes to less than five percent of all cases [1].

The article "Functional Mitral Stenosis Resulting in Recurrent Flash Pulmonary Edema: A Case Report of an Atypical Complication of Streptococcus viridans Endocarditis" was published in 2023. Journal: Cureus.

The pathophysiology of IE requires injury to the endocardium. This initial insult can be secondary to turbulent blood flow, direct mechanical trauma from catheterization, or from preexisting congenital or acquired cardiac lesions such as prosthetic valves. The damaged endocardium serves as a site of platelet and fibrin aggregation resulting in the formation of a sterile vegetation. Subsequent bacteremia, as can be seen following manipulation of the gingiva during dental procedures as in our patient, can result in colonization of these vegetations or direct infection of the damaged endocardium. 

Several microorganisms are associated with IE, with 80% to 90% of cases attributed to gram-positive *Streptococci*, *Staphylococci*, and *Enterococci* organisms [1]. *S. viridans*, as seen in our patient, is the most common cause of subacute IE. The HACEK (*Haemophilus*, *Aggregatibacter*, *Cardiobacterium*, *Eikenella*, *Kingella*) organisms are a group of gram-negative bacteria that colonize the oropharynx and are responsible for one to six percent of all IE cases [1]. Fungal infections, specifically *Candida* and *Aspergillus*, account for approximately one percent of IE cases and are associated with poorer outcomes [1].

A high index of suspicion is needed to diagnose IE as it can present with a wide variety of clinical signs and symptoms. Patients with acute IE typically present with a fever, prompting early infectious work-up with blood cultures. If left untreated, acute IE can progress to rapid destruction of cardiac structures and death within weeks [3]. Subacute IE, as seen in our patient, often presents with a more indolent clinical course. Patients present with a constellation of nonspecific symptoms, including fever, rigors, malaise, night sweats, anorexia, and weight loss leading to delays in diagnosis [3]. It is often not until a complication of subacute IE (such as a major embolic event or structural damage leading to symptoms) presents that clinicians are able to reach a diagnosis. In the case of our patient, a diagnosis of IE was not established until after structural damage to the mitral valve had already occurred.

It is also important to note that the empiric ceftriaxone our patient received earlier in her admission was intended to treat community-acquired pneumonia and was, therefore, only given for five days. Although it would have adequately treated the S. viridans based on susceptibilities, the initial duration of treatment fell well short of the six weeks typically required to treat IE. This may explain why her initial blood cultures were negative, but subsequent blood cultures drawn after completion of the empiric ceftriaxone resulted in positive. 

The article "Functional Mitral Stenosis Resulting in Recurrent Flash Pulmonary Edema: A Case Report of an Atypical Complication of Streptococcus viridans Endocarditis" was published in 2023. Journal: Cureus.

Modern diagnostic criteria for IE involve positive blood cultures, echocardiography, and the modified Duke criteria. Either positive pathological criteria or a combination of major and minor clinical criteria must be met in order to definitively confirm a diagnosis of IE by the modified Duke criteria [2]. It is worth mentioning that the most recent modified Duke criteria specifically mentions new valvular regurgitation, but not valvular stenosis, as a major clinical criterion [2]. Our case highlights some of the limitations of the modified Duke criteria. Our patient did not meet the required major and minor clinical criteria for IE but had pathological confirmation of IE on biopsy. Once the diagnosis of IE is made, treatment consists of antibiotics and possibly surgery. A multidisciplinary approach involving Infectious Disease, Cardiology, and Cardiothoracic Surgery is recommended.

Most complications of IE involve either embolization or damage to cardiac structures [4]. Embolization has been reported in 13% to 44% of patients with IE [4]. Depending on the location, embolization from IE can result in stroke, paralysis, ischemia of the extremities, splenic or renal infarction, pulmonary embolism, and/or abscesses. As a general rule, left-sided vegetations typically result in systemic emboli, whereas right-sided vegetations result in pulmonary emboli. The most common complications of IE are cardiac complications resulting from structural damage, with heart failure being the most common cause of death [4]. Valvular damage resulting in valvular insufficiency and subsequent regurgitation is the most common etiology of IE-associated heart failure. An extensive literature search resulted in few documented cases of functional mitral stenosis as the cause of heart failure in IE [5-7]. Most of these cases involved fungal organisms, not bacterial, as seen in our patient [7]. At present, bacterial endocarditis causing functional mitral stenosis remains a rare condition that has only been described a handful of times in literature. Our case highlights these phenomena, illustrating an atypical presentation of an already uncommon disease process.

## Conclusions

Infective endocarditis is a leading cause of morbidity and mortality in modern medicine. Early detection and treatment are key to improving outcomes. Delays in diagnosis can lead to permanent damage to cardiac structures. Valvular stenosis is a rare late complication of infective endocarditis, which presents with signs and symptoms consistent with heart failure.
